# An Early Warning Intelligent Algorithm System for Forest Resource Management and Monitoring

This article has been retracted.

**DOI:** 10.1155/2022/4250462

**Published:** 2022-10-11

**Authors:** Liheng He, Tingru Zhu, Meng Lv

**Affiliations:** College of Civil Engineering, Nanjing Forestry University, Nanjing 210037, China

## Abstract

The development of remote sensing technology has passed an effective means for forest resource management and monitoring, but remote sensing technology is limited by sensor hardware equipment, and the quality of remote sensing image data is low, which is difficult to meet the needs of forest resource change monitoring. This paper presents a remote sensing image classification method based on the combination of the SSIF algorithm and wavelet denoising. Forest information is extracted from PALSAR/PALSAR-2 radar remote sensing data. The forest distribution map is generated by pixel level fusion algorithm, and the accuracy of the forest distribution map is evaluated by a confusion matrix. The remote sensing image is spatio-temporal fused by the SSIF algorithm to capture more details of forest distribution. The simulation analysis shows that the overall accuracy of the forest classification results obtained by the fusion algorithm is 96% ± 1, and the kappa coefficient is 0.66. The accuracy of forest recognition meets the requirements.

## 1. Introduction

Forest resources are natural resources with the largest land area, the widest distribution, the most complex components, and the most perfect functions. They are also the main body of the terrestrial ecosystem. They play an irreplaceable role in maintaining species diversity, storing carbon, storing water, providing biological resources, and maintaining ecological balance. Forest resources are affected by natural or non-natural factors, and their area, quality, and function are constantly changing. It is a dynamic renewable resource. Accurately grasping the growth and decline of forest resources is the premise of strengthening the construction of a national ecological civilization, and it is also a necessary measure to maintain the sustainable development of the social economy. The traditional forest resources monitoring method based on the artificial ground investigation has the problems of a heavy workload, high cost, long time-consuming, and low efficiency, which is difficult to meet the current needs of forest resources change monitoring. Remote sensing technology has the advantages of detecting a wide range of the ground, obtaining ground information quickly, and being less restricted by the ground. It can quickly reflect the real terrain and landform, and can effectively save human and material resources. It has become one of the important means to quickly obtain information in the current forest resource change monitoring [1, 2]. Nowadays, with the rapid development of remote sensing technology, high spatial resolution remote sensing images can better capture the subtle changes of forest resources in the monitoring of forest resources change, which is conducive to the accurate monitoring of forest resources. It is generally considered to be the most important data source for forest resources change monitoring.

## 2. Literature Review

With the continuous development and innovation of information technology architecture, forest resource dynamic monitoring technology has also gradually developed. With the support of various technologies and years of development, forest resource monitoring and management technology has continuously achieved remarkable results in forestry. Forest resources are constantly changing with the passage of time and have timeliness and variability. The traditional forest resources investigation and monitoring methods can not fully and effectively monitor forest resources. In terms of technology operation and management, it is difficult to meet the current needs of forestry information monitoring and management. With the continuous innovation and integration of forest resource information management technology and forest resource monitoring technology, relevant forestry departments and forestry research institutes have used computer technology to develop and implement forest resource management system and monitoring system, providing support for forest resource management. At present, the information technology of forest resources has been continuously developed. GIS, RS, and GPS technologies are used to comprehensively reform and adjust the forest resources monitoring system, realize the timely, accurate, and efficient monitoring of forest resources, update the forest resources database, and realize the dynamic adjustment and update of forest resources monitoring [3].

In the forest resources monitoring system, the relevant satellite data are used to conduct a comprehensive remote sensing monitoring experiment on the resources of forestry areas. The space and aviation remote sensing monitoring platform is used to monitor and investigate the ground in combination with GIS technology and GPS, and the distribution type, area, and land type of forest resources are checked. In the middle and late stage, the use of 3S technology in forest resources research institutes, forestry experimental bases, and other places across the country has achieved certain results in the monitoring and management of forest resources, but further development is needed. For the application of 3S technology in forest resources monitoring, relevant scholars and researchers proposed that the actual application of monitoring and the experimental methods of operation should be continuously improved to achieve real-time, efficient, and accurate monitoring of forest resources and provide practical methods for forestry management and relevant departments [4]. With the continuous development of science and technology, remote sensing technology has played an important role in the monitoring of forest resource changes. Remote sensing technologies, such as aerospace and aviation, have shown the advantages of traditional monitoring methods in the monitoring of forest resource changes from the accuracy, timeliness, and coverage of operations. The characteristics of its space technology, such as multiplatform, multiangle, multisensor, high resolution, and hyperspectral, make the remote sensing image technology shorten the monitoring cycle time than the traditional monitoring technology in the monitoring of forest resource changes, and solve the shortcomings of forest resource data update difficulties, forest resource monitoring data lack of spatial distribution information and so on. The scope of forest resources monitoring has been expanded, the processing efficiency of the work has been improved, and the current situation and past changes of forest resources have been grasped in time. As a powerful tool for forest resource management and data processing, GIS makes up for many deficiencies of traditional forest resource management and monitoring in data updating, data transmission, and data processing. For example, the huge amount of redundant data, the timeliness of forest resource data, and the integration and updating of forest resource data and remote sensing graphic data. However, due to the rapid development of GIS in the later stage, it has been widely used in forestry, agriculture, forest resources monitoring and investigation, urban planning, military deployment, and other fields. In the application of forest resources management, there are mainly forest resources management information system, forest resources auxiliary decision-making system based on GIS, forest fire prevention system, and so on [5, 6].

## 3. Forest Information Extraction Based on PAL SAR Image

### 3.1. GEE Remote Sensing Cloud Computing Platform

Use JavaScript API to write functions to calculate and process Landsat and Pallar/Pallar-2 remote sensing big data stored in GEE on a high-performance cluster server. The data in PALSAR and PALSAR-2 active microwave sensors are used to extract forest information. Its L-band frequency not only has stronger penetration but also is not affected by the alternation of day and night, cloud shadow, and bad weather. It can realize the Earth observation day and night throughout the day, so as to obtain the information of forest vertical structure. Therefore, it is widely used in forest information extraction and other fields. As shown in Table 1, PALSAR and PALSAR-2 sensors have three different observation modes, so they can observe a wider ground width than ordinary radar sensors [7].

### 3.2. Index Parameter Processing Method

In this study, the annual mosaic data of 2007–2010 and 2015–2021 with a spatial resolution of 25 m from PALSAR-2 sensors covering all the three northern regions are selected. Among them, the annual mosaic data from 2007 to 2010 is from the PALSAR sensor, and the annual mosaic data from 2015 to 2021 is from the PALSAR-2 sensor. Polarization signals based on radar remote sensing image data can be transmitted and received in horizontal and vertical dimensions through L-band, including the HH polarization band in which microwave energy is transmitted and received by radar antenna in the horizontal dimension, and the HV polarization band in which microwave energy is transmitted by radar antenna in the horizontal dimension and received in vertical dimension [8, 9]. In order to reduce the influence of terrain on Earth observation and the distortion of geometric angle, this study uses the 90 m Space Shuttle Radar terrain mission (SRTM) digital elevation model (DEM) to carry out slope correction and orthogonal correction on the backscattering coefficients of HH and HV polarization bands, with a geometric accuracy of about 12 M. The resulting PALSAR/PALSAR-2 mosaic data set includes HH and HV polarized backscatter data, local incident angle and mask information. The size of a pixel is about 25 m × 25 m.

As shown in formula (1), based on the GEE cloud computing platform, for the corrected mosaic data of pallar/pallar-2 in the three north project area, the HH and HV polarization band amplitude data stored in 16 bit digital (DN) form are converted into backscattering coefficients in decibels (DB) pixel by pixel using the calibration coefficient from JAXA:

(1) $$\begin{array}{c} \gamma^{0}\left(dB\right)10\;\log_{10}\;DN^{2}+CF\text{.} \end{array}$$

Here, *γ*^*o*^ (DB) is the converted backscattering coefficient in dB, DN is the amplitude data of HH or HV polarization bands stored in 16 bit digital form, and CF is the absolute calibration coefficient from JAXA, with a value of −83. In addition, because the ratio value and difference value of HH and HV polarization bands are of great significance for extracting land use information, this study calculates the difference value difference (HH-HV) and ratio CHH/HV of the converted HH and HV band backscattering coefficients pixel by pixel through GEE cloud computing platform [10].

(2) $$\begin{array}{c} Difference=HH-HV\text{,} \end{array}$$

(3) $$\begin{array}{c} Ratio=\frac{HH}{HV}\text{.} \end{array}$$

In formulas (2) and (3), HH represents the backscattering coefficient of the transmission and reception of the radar antenna in the horizontal dimension, and HV represents the backscattering coefficient of the transmission and reception of the radar antenna in the horizontal dimension and the vertical dimension. After pixel by pixel calculation and processing of the PAL/pal-2 mosaic data in the three northern regions on the GEE cloud computing platform, we obtained the PAL/pal-2 data with four bands of HH, HV, difference value, and ratio [11, 12].

### 3.3. Decision Tree Classification Algorithm to Extract Forest Information

By calculating the frequency distributions of HH, HV, difference value (HH-HV) and ratio value (HH/HV) of four typical land cover types (forest, water, farmland, and urban land) in the three northern regions, the threshold value of extracting forest distribution information using PALSAR/PALSAR-2 radar remote sensing data is determined. First of all, we collected and visually interpreted 1722 sample points in the three north region using Google Earth's ultrahigh resolution images as a training sample set, called regions of interest (ROI), including 469 forest samples, 432 farmland samples, 429 urban land samples, and 392 water samples. Then, the obtained samples are imported into assets of the GEE cloud computing platform in the form of ShapeFile for analysis, and the annual mosaic data set of PALSAR/PALSAR-2 is imported by using the data resource library in Gee, and the backscatter coefficient is converted pixel by pixel. Then, the HH, HV, HH-HV difference values, and HH/HV ratio values are calculated and used as four bands. Next, the values of the four bands calculated are assigned to the verification sample points one by one, and the results return 1722 sets of characteristic values of samples of interest. Finally, the frequency histograms of HH, HV, difference value (HH-HV), and ratio value (HH/HV) of four typical land cover types are generated, as shown in Figures 1(a)–1(d).

By comparing HH, HV, difference value (HH-HV), and ratio value (HH/HV) of common land cover types, the threshold value of extracting forest information based on PALSAR/PALSAR-2 data in this study is determined [13, 14]. In order to make the classification threshold more reliable, we exclude 2.5% pixels with maximum and minimum backscattering coefficients in HH, HV, HH-HV, and HH/HV and determine the decision tree classification threshold for extracting forest information according to the 95% confidence interval.

As shown in Figure 1, from the frequency histogram of HH and HV backscattering coefficients, it can be seen that the HH and HV values of water bodies are significantly lower than those of forests, farmland, and urban land, and there is almost no overlap with forests. This is because the reflecting surface of the water body is relatively smooth, and most of the backscattering can be reflected through specular reflection. Therefore, the water body can be easily distinguished from forests, urban land, and most farmland land cover types by HH or HV backscattering coefficient. Because the L-band of the PALSAR/PALSAR-2 sensor has strong penetration into the forest, the energy emitted when it is incident will interact with the trunk and branches of trees, resulting in a large amount of volume scattering. Therefore, the HH and HV backscattering coefficients of the forest are high, the difference value (HH-HV) is low, and the HV of the farmland is low. Therefore, the forest can be distinguished from most of the farmland. Due to the complex spatial structure of urban land, the backscatter coefficients of HH and HV are high, and HH-HV and HH/HV also overlap with forests to a certain extent. Therefore, only HH, HV, difference value (HH-HV) and ratio value (HH/HV) are not enough to completely distinguish the types of forest and urban land cover. Finally, forests can be distinguished from water bodies, most farmland, and some urban land cover types. Therefore, as shown in formula (4) and Figure 2, this study constructs a decision tree classification threshold for extracting forests:

(4) $$\begin{array}{c} \left(-16<HV<-8\right)AND\left(2<Difference<8\right)AND\left(0.3<Ratio<0.85\right)\text{.} \end{array}$$

Based on the above-given analysis of HH, HV, difference value (HH-HV), and ratio value (HH/HV) backscatter coefficient thresholds of four common land cover types, it can be seen that there are obvious rules for extracting information of different land cover types based on PALSAR/PALSAR-2 radar remote sensing data, which lays a good foundation for building decision trees for classification. Since the focus of this study is the distribution of forests, for the convenience of followup research, we combined the classification results into the forest and nonforest, and generated forest/nonforest distribution maps from 2007 to 2010 and 2015 to 2021, with a spatial resolution of 25 m.

## 4. Spatiotemporal Fusion Algorithm Based on SSIF Learning

### 4.1. Remote Sensing Image Degradation Model

A remote sensing image is a digital image obtained by means of photography, aerial scanning, or microwave imaging by sensors mounted on the remote sensing platform. Its basic unit is pixels, and the gray value of surface information is recorded by the DN value [15]. The superresolution reconstruction of remote sensing image is the process of using a certain conversion model to complement the information of low-resolution images, so as to reconstruct high-resolution images. Assuming that the low resolution image *l* meets a certain degradation relationship with its corresponding high resolution image *h*, the low resolution image *l* can be regarded as the result of a series of degradation processes such as down sampling and blurring of the high resolution image *h*. therefore, the relationship between the two can be established by a remote sensing image degradation model, as shown in relation:

(5) $$\begin{array}{c} L=SBH+n\text{.} \end{array}$$

In (5), *L* is a low resolution image; H is a high-resolution image; *S* is the down sampling matrix; *B* represents fuzzy process; *N* is the noise generated when *H* is converted to *L*.

The super-resolution reconstruction of remote sensing image is the inverse process of the degradation model of remote sensing image, which needs to introduce a priori knowledge to solve. At present, sparse representation theory is one of the most effective methods.

#### 4.1.1. Sparse Representation Principle of Remote Sensing Image

Sparse representation theory originated in the field of signal processing. Its main purpose is to use as few atoms as possible to approximate the original signal from a given super complete dictionary, so as to more refine the information contained in the signal. In recent years, the sparse representation method is mainly used in remote sensing image processing. Relevant research shows that most remote sensing images can be sparse representation because of their relevance and redundancy [16]. The sparse representation model of remote sensing image is shown in the following equation:

(6) $$\begin{array}{c} \min{\left\|a\right\|}_{0}s.t.X=D\times a\text{.} \end{array}$$

According to the above-given sparse representation theory, the sparse representation of image *x* can be obtained from a suitable over a complete dictionary, and in the process of sparse representation, image *x* should be approximately represented with as few atoms as possible. It can also be understood that the sparse representation coefficient a is mostly equal to or close to 0, that is, assuming that a contains *f* nonzero terms, which meets the condition *f* < *n* < *k*. In order to measure the number of nonzero elements in the sparse coefficient a, *l* is usually used. Norm is expressed. Theoretically, *l* is solved in equation. Norm is the simplest sparse measure, but *l* is used. Norm regularization to achieve sparseness is a NP hard (non determined polynomial hard) problem, so equation (7) is often transformed into the following equation:

(7) $$\begin{array}{c} \min{\left\|a\right\|}_{1}s.t.{\left\|X-Da\right\|}_{2}^{2}<\varepsilon \text{.} \end{array}$$

By introducing a Lagrange multiplier, (7) can be further optimized into an unconstrained optimization problem:

(8) $$\begin{array}{c} \min{\left\|X-Da\right\|}_{2}^{2}+\gamma {\left\|a\right\|}_{1}\text{.} \end{array}$$

In (8), *γ* is a Lagrange multiplier, which can mediate the fidelity of the image and the sparsity of the sparse coefficient. The more 0 elements of a, the better the sparsity.

It can be concluded that there are two optimization variables in sparse representation, dictionary D and sparse coefficient a. The solution to this optimization problem is generally to fix one optimization variable first, then optimize the other variable, and finally proceed alternately. At present, the sparse coefficient solving algorithm can be divided into a greedy algorithm and convex optimization based algorithm. According to the relevant literature, the greedy algorithm has better performance than the convex optimization algorithm, so greedy algorithm is often used for sparse coding [17].

#### 4.1.2. Dictionary Construction

K-SVD (k-singular value decomposition) dictionary learning algorithm is a derivative algorithm of k-means. According to the principle of minimum error, the algorithm decomposes the error term E and through SVD, selects the decomposition term with minimum error to update the dictionary and sparse representation coefficient, and finally obtains the optimal solution through the process of alternating iteration. The specific steps of the K-SVD dictionary learning algorithm are as follows:

(1) Randomly select *k* column vectors from the original sample, initialize dictionary D, normalize all column vectors, and set the number of iterations *r*
(2) Fix the dictionary D, and use the OMP algorithm to solve the sparse representation coefficient of each training sample
  (9) $$\begin{array}{c} a_{i}=\underset{D_{r-1,x}}{argmin}{\left\|X-D_{r-1}\alpha_{i}\right\|}_{F}^{2}s.t.\left\|X\right\|\leq F,i=1,2,\cdots ,k\text{.} \end{array}$$
(3) Update the dictionary D obtained in step (2) atom by atom and then use formula (9) to perform singular value decomposition (SVD) on the error matrix to extract the most important features in the matrix
  (10) $$\begin{array}{c} E_{k}=U\Delta V^{T}\text{.} \end{array}$$
(4) The dictionary D and the sparse representation coefficient are iteratively updated until the final dictionary is obtained

The main task of super-resolution reconstruction based on the principle of sparse representation is to use the method based on sparse representation to obtain the relationship between images with different spatial resolutions, so as to complete the prediction and construction of high-resolution images at another time. Therefore, it is necessary to establish high-resolution and low-resolution dictionaries under the feature blocks of high-resolution and low-resolution images (relatively high and low), and establish the relationship between them. In the process of dictionary construction, if the image blocks corresponding to the high and low resolution images are sampled at the same time, the resulting high and low resolution dictionary also meets the remote sensing image degradation model, and the expression (11) can be obtained:

(11) $$\begin{array}{c} DL=SBD_{H}+n. \end{array}$$

By introducing (11) into the sparse representation model of remote sensing images, we can get the following equation:

(12) $$\begin{array}{c} X_{L}=SBD_{H}\times \alpha +n_{1}\text{.} \end{array}$$

(12) is a low resolution image, which can be obtained in the same way:

(13) $$\begin{array}{c} X_{H}=SBD_{H}\times \alpha +n_{2}\text{.} \end{array}$$

According to the observation formulas (12) and (13), images *X*_c_ and *X*_H_ with different spatial resolutions have the same sparse representation coefficient a in the process of super-resolution reconstruction based on sparse representation, so we can use the same sparse representation coefficient a as a bridge from low resolution remote sensing image to high-resolution remote sensing image reconstruction to realize super-resolution reconstruction [18, 19].

### 4.2. Sparse Spatio-Temporal Fusion Algorithm Based on Single Pair of Images

The image data used by SSIF algorithm is consistent with that of starm algorithm. Landsat Image at time to, MODIS Image and MODIS Image at time TK are the data sources. Considering the large spatial resolution difference between Landsat Image (high resolution image) and MODIS Image (low resolution image), if the two images are directly fused, it will lead to a huge prediction error. The way to solve this problem is to improve the spatial resolution of the MODIS Image and then integrate the MODIS Image with the original Landsat Image. Through the idea of the remote sensing image degradation model, it is assumed that MODIS Image (corresponding band) is the result of Landsat image degradation through a series of down sampling, blurring, and other processes. Considering the upper limit of super-resolution reconstruction, the spatial resolution of MODIS Image at time to and TK is improved and reconstructed into a transition image with spatial resolution between MODIS and Landsat Image by using the super-resolution reconstruction principle based on sparse representation, and then the information of transition image and Landsat Image is collected by using high pass filtering, so as to generate Landsat Image at prediction time TK [20].

Suppose that Landsat Image and MODIS Image at time t0 are l0 and M0 respectively; The Modsi image at TK time is MK; The generated transition images are t0 and TK respectively. The super-resolution reconstruction of the MODIS image includes two steps, that is, using the known M0 and l0 to establish the dictionary training set, and then complete the construction of the transition image. The specific steps are as follows.

#### 4.2.1. High and Low Resolution Dictionary Training

Obtain the high-resolution features (feature blocks extracted from the difference image of l0-m0) and low-resolution features (feature blocks of M0) of MODIS Image and Landsat Image at time T0, list the two feature blocks, input them into the K-S VD dictionary training model, and obtain the low-resolution Dictionary:

(14) $$\begin{array}{c} \left\{D_{L},\Lambda^{*}\right\}=\underset{D_{L,\Lambda }}{argmin}\left\{{\left\|x-D_{L},\Lambda^{*}\right\|}_{F}^{2}\right\}s.t.\forall_{i},{\left\|\alpha_{i}\right\|}_{0}\leq K_{0}\text{.} \end{array}$$

In equation (14), *X* is the sampling matrix after the serialization of MODIS gradient image feature blocks, *n* is the sparse coefficient of each column corresponding to *x*, where the given sparse coefficient *n*^∗^ is a nonsingular matrix, and DL is the obtained low resolution dictionary. Since the high-resolution dictionary and the low-resolution dictionary have the same sparse representation coefficient, the corresponding high-resolution dictionary training can be carried out with the following equation:

(15) $$\begin{array}{c} D_{G}=\underset{D_{G}}{argmin}\left\{{\left\|Y-D_{L},\Lambda^{*}\right\|}_{F}^{2}\right\}\text{.} \end{array}$$

Equation (15) needs to be solved by using the generalized inverse matrix of the following equation:

(16) $$\begin{array}{c} D_{G}=Y{\left(\Lambda^{*}\right)}^{+}=Y\Lambda^{*t}{\left(\Lambda *\Lambda^{*T}\right)}^{-1}\text{.} \end{array}$$

#### 4.2.2. Transition Image Construction

After the dictionary training, it is used to construct the transition image. The transition prediction image *T*_K_ is generated based on the MODIS Image *M*_K_ at *T*_K_ time. First, the gradient feature image block of *M*_K_ is sampled in the same way as in dictionary training, assuming that the ith column of *X*_K_ is *X*_K_; the OMP algorithm in greedy algorithm can solve the sparse coefficient matrix of its corresponding low resolution dictionary DL, so as to obtain the one-to-one corresponding sparse coefficient matrix *A*_I_ in each low resolution image block. Based on the principle of sparse representation, using the sparse coefficient *A*_K_ of MODIS Image (*M*_O_) at *T*_K_ time and the high-resolution dictionary aligned at *t*_0_ time, the difference image *Y*_K_ of high-resolution and low-resolution images at *T*_K_ time can be obtained, and finally the transition prediction image *T*_K_ can be obtained. Similarly, the transition prediction image *t*_0_ at *t*_0_ time can be obtained.

#### 4.2.3. High Pass Filtering

Since the difference image between Landsat Image and MODIS Image at t0 time for dictionary training has a high degree of similarity in phenological changes and changes in surface coverage types, assuming that the transition prediction image t0 and TK obey the linear change relationship, the following linear transformation model can be obtained:

(17) $$\begin{array}{c} T_{k}=a\times T_{0}+b\text{,} \end{array}$$

(18) $$\begin{array}{c} L_{k}=a\times L_{0}+b\text{.} \end{array}$$

The solution formula of Landsat Image at *T*_*K*_ time can be derived from (17) and (18):

(19) $$\begin{array}{c} L_{k}=T_{k}+\frac{T_{k}}{T_{0}}\times \left(L_{0}-T_{0}\right)\text{.} \end{array}$$

### 4.3. Forest Resource Change Monitoring with High Spatial Resolution Fusion Images

#### 4.3.1. Establishment of Classification System

Before the classification of remote sensing images, it is necessary to establish a classification system according to the information contained in the images of the study area and the purpose of the study. According to the classification of land use status and the main technical provisions for the planning, design, and investigation of forest resources, the classification standards of forest land are shown in Table 2. The classification system is formulated according to the macro situation of national forest land and forest resources.

Forest resources are the general name of forest land and the forest organisms it grows, and forest land resources are the main body of forest resources. The forest resources referred to in this paper are aimed at forest land resources. Considering that there are still some differences between the high spatial resolution fusion image and the actual GF-2 MSS image, and the insufficient characteristics of the 4 m spatial resolution GF-2 MSS image, the recognition ability of forest land types is limited, so it is difficult to make a fine distinction. Therefore, the shrub land, sparse forest land, and forest land in the study area are collectively referred to as forest land in this paper. Nonforest land is divided into construction land, cultivated land, water body, and unused land, among which residential areas, urban roads, and other construction land are collectively referred to as construction land.

#### 4.3.2. Classification Feature Information Extraction

The purpose of feature information extraction is to represent all the information of the image with the least and most significant features, and improve the discrimination between different ground objects while reducing the dimension, so as to distinguish the ground types to the greatest extent.

*(1) Spectral Characteristics*. In this paper, four bands of red, green, blue, and near infrared of GF-2 MSS image on January 16, 2021, and high spatial resolution fusion image on October 9, 2021, generated by SIF algorithm are selected as spectral characteristic variables to participate in classification.

*(2) Texture Features*. In this paper, the co-occurrence measures texture analysis tool in ENVI 5.3 software is used to calculate the gray level co-occurrence matrix of the first principal component and the second principal component after the principal component transformation. The 7 × 7 base window is used respectively, and the gray quantization level is set to 64 to extract the texture features. This paper selects three texture features: contrast, variance and mean as auxiliary feature information of image classification.

*(3) Vegetation Index*. Vegetation index is an effective index to measure the status of surface vegetation. This kind of index combines images and different bands (often referred to as visible light, red band, and near-infrared band) in a linear or nonlinear way to enhance the vegetation characteristic information. Among them, normalized vegetation index and ratio vegetation index are two commonly used vegetation indexes. Both of them make use of the characteristics of vegetation with strong absorption ability in the red light band and strong reflection ability in the near-infrared band to calculate the band of the near-infrared band and the red light band [21].

Normalized vegetation index (NDVI) is to normalize the red light band and near-infrared band to enhance vegetation information. The index is between [−1, 1]. When the value of NDVI is greater than 0, it indicates that there is vegetation cover on the ground; When NDVI value is less than or equal to 0, it means that the surface is not covered by vegetation or the surface is covered by nonforest land such as clouds, water or snow. In short, the NDVI index can enhance the differentiation between forest land and nonforest land.

The ratio vegetation index (RVI) is the division of near-infrared band and visible red band to enhance vegetation information, which is consistent with the concept of normalized vegetation index. Generally speaking, the RVI value of a healthy green vegetation covered area is much greater than 1, and when the RVI value is near 1, it means that there is no vegetation cover or the vegetation coverage is low in this area.

*(4) Normalized Water Index*. There is a large area of water in this study area. In order to increase the contrast between water and forest land and between water and other land types, normalized difference water index (NDWI) is often used. Because the spectral corresponding curve of the water body decreases from the green light band to the infrared band, while the spectral corresponding curve of vegetation is on the contrary, this index can not only highlight the characteristic information of the water body but also weaken the characteristic information of soil and vegetation. The classification feature parameters extracted in this paper are shown in Table 3. The study area is classified according to the following feature parameter set.

#### 4.3.3. Image Adaptive Appendix Wavelet Denoising

Signals are usually divided into high-frequency and low-frequency signals, in which low-frequency signals contain useful information in a large range and large scale of the image, while high-frequency signals reflect the edge and detail information of the image, and it is also the location of noise concentration. According to the relevant research, wavelet denoising benefits from its multiresolution, low entropy, decorrelation, flexibility of base selection, and other characteristics and can effectively remove the noise in remote sensing images. As shown in Figure 3, taking the noisy signal Sn as the input, first complete the wavelet decomposition of the signal, that is, the low-frequency and high-frequency signals in the input signal Sn are separated, and then the decomposed high-frequency coefficients are threshold quantized according to the relevant theory of the selected threshold method. Finally, the processed wavelet coefficients are used for the inverse wavelet transform to complete the signal reconstruction to obtain the denoised signal.

### 4.4. Comparison and Analysis of Simulation Results

#### 4.4.1. Accuracy Analysis

The accuracy evaluation of classification results is a measure of the reliability of classification results, and the confusion matrix is the standard form of accuracy evaluation. The confusion matrix is a comparison matrix obtained by calculating the pixels of the classification data set and the verification data set, which is used to verify whether the classification of the classification data set and the verification data set at the corresponding position are consistent, so as to obtain the classification accuracy of the image. In this paper, the GF-2MSS images on January 16, 2021, and October 9, 2021, are randomly sampled by visual interpretation method. As the real samples, the validation sample data set is constructed. Finally, the classification accuracy of the images is evaluated by the calculation results of the confusion matrix.

Table 4 shows the classification confusion matrix of GF-2 MSS image classification feature set on January 16, 2021, in which the overall classification accuracy of random forest classification is 84.42%, kappa coefficient is 0.81, the overall classification accuracy of adaptive threshold wavelet denoising + random forest classification is 89.92%, kappa coefficient is 0.87, and the overall accuracy of adaptive threshold wavelet denoising + random forest classification method is 5.5% higher than that of random forest classification method. Kappa coefficient increased by 0.06.

According to Table 5, the user accuracy and mapping accuracy of various ground objects in random forest classification are higher than 75%, of which the classification accuracy of water and forest land is higher than 88%, but the classification accuracy of cultivated land and unused land is low, because some cultivated land has low vegetation coverage, and its spectral response curve is similar to that of unused land, which makes it difficult to distinguish them. The areas with high vegetation coverage are close to the reflectance of forest land, which is easy to produce misclassification. In addition, the generation process of remote sensing images will be affected by uncertain factors, resulting in “abnormal points,” so there is also the possibility of misclassification. The classification method combining adaptive threshold wavelet denoising and random forest has improved the mapping accuracy and user accuracy of cultivated land, unused land, construction land, forest land, and water body. Among them, the mapping accuracy of cultivated land, construction land, forest land, and unused land has been improved by 7.25%, 9.52%, 2.22%, and 6.64%, respectively, and the user accuracy has been improved by 8.02%, 3.42%, 8.23%, and 6.32%. Due to the large spectral difference between water body and other ground objects and high discrimination, the accuracy improvement is small.

Table 6 shows the classification confusion matrix of the classification feature set of high spatial resolution fusion images on October 9, 2021, in which the overall accuracy of random forest classification is 81.4%, and the kappa coefficient is 0.85. The overall classification accuracy of adaptive threshold wavelet denoising + random forest classification is 84.83%, and the kappa coefficient is 0.89. Compared with the random forest classification method, the overall accuracy of the adaptive threshold wavelet denoising + random forest classification method is improved by 3.43%, and the kappa coefficient is improved by 0.04. Combined with Table 7, the adaptive closed-value wavelet denoising + random forest classification method has better improved the mapping accuracy and user accuracy of cultivated land, forest land, unused land, and water, but the user accuracy of construction land has been reduced by 1.81%.

#### 4.4.2. Monitoring Results of Forest Resource Change

In order to obtain the increase and decrease of the number and distribution of forest land after mutual transformation with other land types, and then obtain the change of forest resources in this region, nonforest land is not the research object of this paper, so this paper does not discuss the change between nonforest land. Using the postclassification comparison method to monitor the changes of the two images, the thematic map of forest resource cover change in the study area can be obtained. According to the thematic map of forest resource cover change in the study area, the spatial location information and the direction information of forest land change in the study area can be obtained. The areas of forest land change in the study area are distributed on both sides of the river, and there are many changes with cultivated land and unused land. In order to further obtain the change area of forest land and the change rate between forest land and nonforest land, use ENVI software to calculate the transfer matrix based on the change results of forest resource coverage, and the statistical results are shown in Table 8 and Figure 4.

According to Table 8 and Figure 4, from January to October 2021, the area of forest land turned into unused land was 468496 m^2^, with a change rate of 0.94%, the area of forest land turned into cultivated land was 1339424 m, with a change rate of 2.78%, the area of forest land turned into the water was 19632 m^2^, with a change rate of 0.04%, the area of forest land turned into construction land was 306640 m^2^, with a change rate of 0.64%, and the total reduced area of forest land was 2134192 m^2^. The area from unused land to forest land is 525520 m^2^, with a change rate of 1.09%, the area from cultivated land to forest land is 860120 m^2^, with a change rate of 1.79%, the area from water to forest land is 66768 m^2^, with a change rate of 0.14%, the area from construction land to forest land is 24784 m^2^, with a change rate of 0.050/a, and the total increased area of forest land is 1477192 m^2^. In general, from January to October 2021, the forest area in the study area decreased by 657000 m^2^, that is, the forest coverage decreased by 1.36%, and the forest resources decreased.

## 5. Conclusion

The process and accuracy evaluation of optical remote sensing data Landsat and radar remote sensing data PALSAR/PALSAR-2 fusion algorithm are introduced. Firstly, the nearest neighbor algorithm is used to adjust the spatial resolution of the forest information extracted from the two remote sensing data sources, and then the appropriate fusion method is used to fuse to generate the final forest distribution map. Next, taking the interannual and intra-annual vegetation index time series generated from Google Earth ultrahigh resolution images and Landsat and MODIS images from collect Earth as reference data, the accuracy of the forest distribution map obtained by the fusion algorithm is evaluated based on the validation sample data set, and compared qualitatively and quantitatively with the four mainstream medium and high spatial resolution forest distribution maps in the market. The forest distribution map obtained in this study has the highest overall accuracy of 96% ± 1% and kappa coefficient of 0.66. In addition, this chapter analyzes the reasons why the classification results of the fusion algorithm are inconsistent with other forest distribution maps from the two aspects of forest definition and data source.

This paper introduces the basic principle of the SSIF algorithm, and then expounds on the principle of remote sensing image degradation model, sparse representation principle, dictionary construction principle, and super-resolution reconstruction principle based on sparse representation theory related to the SSIF algorithm. Finally, the spatio-temporal fusion framework of the Landsat 8 OLI image and GF-2 MSS image of the SSIF algorithm is established respectively, and the spatio-temporal fusion of the Landsat 8 OLI image and GF-2 MSS image is completed. Because continuous time series GF-2mss image data and Landsat 8 OLI image data are difficult to obtain, this paper only considers the spatio-temporal fusion of single temporal medium and high spatial resolution remote sensing images.

The classification method based on adaptive closed value wavelet denoising and random forest can better reduce the “salt and pepper noise” generated by image classification. This is because adaptive threshold wavelet denoising removes some high-frequency components in the image on the basis of retaining the original spectral information of the image, so as to suppress the “noise” in the image, reduce the uncertainty factors in the image classification process, and further improve the classification accuracy of the image. It shows that the classification method based on adaptive closed value wavelet denoising and the random forest is feasible.

## Figures and Tables

**Figure 1:** Frequency histogram of backscattering coefficients of four typical land cover types.

**Figure 2:** Decision tree classification based on PALSAR/PALSAR-2 radar remote sensing data.

**Figure 3:** Wavelet threshold denoising process.

**Figure 4:** Change rate of forest resources.

**Table 1:** Data specification of PALSAR/PALSAR-2 sensor.

Observation mode	High resolution		Scanning synthetic aperture	Polarization
Center frequency	1270 MHz (L-band)			
Chirp bandwidth	28 MHz	l4 MHz	14 MHz, 28 MHz	14 MHz
Polarization mode	HH/VV	HH + HV/VV + VH	HH/VV	HH + HV + VH + VV
Incident angle	8 to 60°	8 to 60°	18 to 43°	8 to 30°
Spatial resolution	7–44 m	14–88 m	100 m (Repeat scan)	24–89 m
Detection width	40–70 km	40–70 km	250–350 km	20–65 km
Bit length	5 bits	5 bits	5 bits	3/5 bits
Data rate	240 Mps	240 Mps	120 Mps, 240 Mps	240 Mps
Working mode	Side view 34.3°		Side view 34.1°	Side angle of view 21.5°

**Table 2:** Forestry land classification standards.

First level	Woodland	Nonforest land
Second level	Forested land	Cultivated land
	Open woodland	Pasture
	Shrub land	Waters
	Immature forest land	Unused land
	Nursery land	Land used for building
	Nonstanding forest land	
	Suitable forest land	
	Land for forestry auxiliary production	

**Table 3:** Statistics of characteristic parameters.

Characteristic information	Characteristic parameter	Number
Spectral information	B, G, R, NIR, NDVI, RVI, NDWI	7
Texture information	PC1 mean, PC1 variance, PC1 contrast, PC2 mean, PC2 variance PC2 contrast	6

**Table 4:** Confusion matrix of GF-2MSS image classification feature set on January 16, 2021.

Category	Random forest					Adaptive threshold wavelet denoising + random forest				
	Cultivated land	Land used for building	Woodland	Unused land	Water body	Cultivated land	Land used for building	Woodland	Unused land	Water body
Cultivated land	321	23	30	44	6	350	9	25	32	5
Land used for building	19	340	9	38	5	20	400	7	30	1
Woodland	34	15	400	12	4	6	10	410	8	2
Unused land	23	41	6	322	10	25	20	8	350	4
Water body	3	1	5	6	400	1	2	3	3	420
	Overall classification accuracy = 84.42% kappa coefficient = 0.81					Overall classification accuracy = 89.42% kappa coefficient = 0.87				

**Table 5:** Classification accuracy statistics of GF-2 MSS image classification feature set on January 16, 2021.

Category	Random forest				Adaptive threshold wavelet denoising + random forest			
	Cartographic accuracy (%)	User accuracy (%)	Misclassification error (%)	Leakage error (%)	Cartographic accuracy (%)	User accuracy (%)	Misclassification error (%)	Leakage error (%)
Cultivated land	80.25	75.71	24.29	19.75	87.50	83.73	16.27	12.50
Land used for building	80.95	83.33	16.67	19.05	90.48	86.76	13.24	9.52
Woodland	88.89	86.02	13.98	11.11	91.11	94.25	5.75	8.89
Unused land	76.30	80.10	19.90	23.70	82.94	86.42	13.58	17.06
Water body	94.91	96.47	3.53	5.09	97.22	98.13	1.87	2.78

**Table 6:** Confusion matrix of classification feature set of high spatial resolution fusion image on October 9, 2021.

Category	Random forest					Adaptive threshold wavelet denoising + random forest				
	Cultivated land	Land used for building	Woodland	Unused land	Water body	Cultivated land	Land used for building	Woodland	Unused land	Water body
Cultivated land	250	23	45	32	25	250	25	15	29	10
Land used for building	12	240	15	14	0	10	400	21	18	2
Woodland	50	10	400	6	5	40	8	410	6	4
Unused land	24	40	2	322	10	28	36	2	350	4
Water body	4	10	3	5	300	2	1	1	4	300
	Overall classification accuracy = 81.4% Kappa coefficient = 0.85					Overall classification accuracy = 84.83% Kappa coefficient = 0.89				

**Table 7:** Classification accuracy statistics of high spatial resolution fusion image classification feature set on October 9, 2021.

Category	Random forest				Adaptive threshold wavelet denoising + random forest			
	Cartographic accuracy (%)	User accuracy (%)	Misclassification error (%)	Leakage error (%)	Cartographic accuracy (%)	User accuracy (%)	Misclassification error (%)	Leakage error (%)
Cultivated land	73.53	64.94	35.06	26.47	76.47	76.47	23.53	23.53
Land used for building	70.00	83.67	16.33	30.00	76.67	81.85	18.15	23.33
Woodland	85.56	84.43	15.57	14.44	91.11	87.61	12.39	8.89
Unused land	82.86	79.23	20.77	17.14	83.71	80.72	19.28	16.29
Water body	87.50	92.72	7.28	12.50	93.75	97.4	2.60	6.25

**Table 8:** Statistical table of forest land changes in the study area from January 2021 to October 2021.

Type of ground feature change	Change area (m^2^)	Rate of change (%)
Forest land—unused land	468496	0.97
Woodland cultivated land	1339424	2.78
Woodland water body	19632	0.04
Forest land—construction land	306640	0.64
Unused land forest land	525520	1.09
Cultivated land forest land	860120	1.79
Water forest	66768	0.14
Construction land—forest land	24784	0.05

## Data Availability

The labeled data set used to support the findings of this study is available from the corresponding author upon request.
